# The Clinical Study of Bladder Flap Ureteroplasty (Psoas Hitch) in the Treatment of Lower Ureteral Injuries and Strictures (19 Cases)

This article has been retracted.

**DOI:** 10.1155/2022/4607735

**Published:** 2022-05-24

**Authors:** Wei Tang, Huiqing Niu, Yunbo Yang, Hui Li, Haichao Liu, Jiaxing Zhang, Peng Zhang

**Affiliations:** Department of Urology, Hebei Yanda Hospital, Langfang City 065201, Hebei Province, China

## Abstract

**Objective:**

The aim of this study was to investigate the efficacy and safety of bladder flap ureteroplasty (psoas hitch) in the treatment of lower ureteral injuries and strictures.

**Methods:**

19 patients with lower ureteral injuries and strictures scheduled for a bladder flap ureteroplasty (psoas hitch) in our hospital from January 2020 to January 2021 were recruited. The outcome measures included treatment efficacy and safety.

**Results:**

The operative time, intraoperative bleeding, catheter extubation time, hospital stay, extubation time of ureteral stent, and follow-up time were (125.36 ± 15.38) min, (75.37 ± 11.09) ml, (7.25 ± 1.04) d, (8.76 ± 1.11) d, (46.34 ± 7.66) d, and(19.27 ± 1.27) months, respectively. No serious perioperative adverse reactions were observed, and all the symptoms of patients were relieved.

**Conclusion:**

Bladder flap ureteroplasty (psoas hitch) is safe and effective for the treatment of lower ureteral injuries, with advantages such as less intraoperative bleeding and trauma and rapid recovery, so it is worthy of promotion. This was a retrospective study supervised by the Ethics Committee of Hebei Yanda Hospital.This trial is registered with no. hebYD076.

## 1. Introduction

The ureter, connecting the kidney and bladder, is the crucial urinary catheter in the body and is vulnerable to damage. The exogenous damage is not frequently seen in the ureter. However, abdominal procedures performed near the ureter may lead to ureteral injuries. Postoperative symptoms such as low back pain, lumbar distension, and fever caused by postoperative infection are unpredictable [1–4]. The common clinical injuries, including stenosis, damage, and necrosis, may be associated with poor urine drainage and subsequent infection or renal dysfunction, seriously compromising the patient's health. Therefore, effective and timely treatment measures are of great significance [5–8]. Ureterocystoplasty with ureteral reflux for patients with unilateral renal tuberculosis and contralateral hydronephrosis has been improved in clinical practice [9–12]. The present study explored the effectiveness and safety of bladder flap ureteroplasty (psoas hitch) in the treatment of lower ureteral injuries and strictures by retrospectively analyzing 19 cases in our hospital.

## 2. Research Process

### 2.1. Ethics Approval and Consent to Participate

Family members of the patient have full understanding of the research process and signed the consent form. This was a retrospective study supervised by the Ethics Committee of Hebei Yanda Hospital (no. hebYD076) with no interference to the treatment process. All the methods were carried out in accordance with the Declaration of Helsinki.

#### 2.1.1. Inclusive Criteria

- Patients met the clinical diagnostic criteria of lower ureteral injuries and strictures, and the diagnosis was confirmed by color doppler ultrasound, intravenous urography, cystoscopy, and computed tomography (CT) of the urinary system.
- The disease was a benign lesion, and there was no contraindication in the preoperative examination.
- With complete clinical data
- The patients and their families have a full understanding of the research process and provided written informed consent

#### 2.1.2. Exclusive Criteria

- With malignant tumors, serious organic diseases, or coagulation disorders
- With renal inadequacies
- In pregnancy or lactation

#### 2.1.3. Patient Screening

19 patients with lower ureteral injuries and strictures scheduled for bladder flap ureteroplasty (psoas hitch) in our hospital from January 2020 to January 2021 were recruited. This was a retrospective study supervised by the ethics committee.

#### 2.1.4. Methods

With the patient in a supine position, corresponding preoperative preparations for laparoscopic pelvic surgery such as endotracheal intubation and general anesthesia were performed. The upper edge of the umbilicus was punctured with a Veress pneumoperitoneum needle, followed by the placement of the laparoscopic lens and a 10 mm Trocar. A 10 mm (affected side) Trocar and a 5 mm (healthy side) Trocar were placed at the lateral edge of bilateral rectus abdominis 3 cm below the umbilicus, and a 5 mm Trocar could be placed 3 cm inside the anterior superior iliac spine based on the actual situation of the patient. The retroperitoneum was opened from the medial side of the affected iliac artery, and iliac vessels were used as anatomical landmarks for the ureter. The free distal ureter was clipped with Hem-O-lock, and the proximal ureter was cut longitudinally for about 1 cm. After freeing the proximal ureter for about 7 cm upward, the bladder wall and Retzius space were separated in a U shape, until the parietal angle of the bladder could be secured with psoas muscle without tension. Psoas muscle was exposed, the bladder wall was pulled to its surface, and the psoas muscle fascia and the seromuscular layer of the bladder were secured using a 2-0 absorbable suture. The pattern of bladder psoas hitch is shown in Figure 1.

The superior and posterior portions of the bladder were freed, on which a 2.5 cm wide flap was made. A guidewire was drawn at the two corners at the end of the flap, and the f16–f18 catheter was wrapped between the bladder flaps, after which they were sutured together, with minimal disruption of the mucosal layer [13, 14]. The catheter was pulled out, and the ureteral catheter or double-J ureteral stent was placed in the proximal ureter, after which was introduced into the bladder through the valve tube. Then, the catheter was guided out of the body through the anterior wall of the bladder and secured, anastomosing the end of the valve tube and the ureteral segment [15, 16]. The bladder wall was sutured after the placement of the cystostomy tube, followed by the placement of the drainage tube. 200 ml of normal saline was injected into the bladder, and the operation was terminated only when there was no exudation.

Patients were given 100 mL of enoxacin injection (Wuhan Yuanda Pharmaceutical Group Co., Ltd., State Drug quantification H10970300, specification 100 mL: 0.2 g) intravenously intraoperatively and postoperatively to prevent infection twice a day. Patients were treated with Shiduqing clear capsules (Guangxi Yulin Pharmaceutical Group Co., Ltd., State Drug Administration Z45021731, specification 0.5 g/capsule) at 3 d before surgery and after postoperative exhaustion. The treatment lasted for 7 d.

#### 2.1.5. Outcome Measures

The patient's age, gender, disease course, pathogenic cause, affected side, and other general information were counted. Their operative duration, intraoperative bleeding, catheter extubation time, hospital stay, extubation time of ureteral stent, follow-up time, and adverse reactions were recorded. The cystography and examination results were collected before and after treatment. The clinical efficacy was evaluated using the results of ultrasound or retrograde imaging of the ureteral recovery of the patients. Markedly effective: the imaging shows complete patency of the ureter and normalization of urinary function, the patients have no discomfort during urination, and clinical symptoms disappear. Effective: the imaging examination shows that the ureter is basically patent, the patient's urinary function is largely unaffected, and most of the patient's symptoms have disappeared. Ineffective: the imaging examination shows an abnormal ureter, with great discomfort and dyspareunia in urination, and no improvement was seen in the disease condition.

#### 2.1.6. Statistical Analysis

The graphics were plotted by GraphPad Prism 7 (GraphPad Software, San Diego, USA). K-S was used to detect the normality distribution of the data. The counting data and measurement data were exhibited as (*n* (%)) and (*x* ± *s*). SPSS 22.0 was used to calculate the diversity of data, and a *P* value of 0.05 or lower was claimed as statistically significant.

## 3. Results

### 3.1. General Information

The age of 19 patients ranged from 19 to 37 years with an average of (26.34 ± 4.51) years. Disease courses were 3–8 months with a mean of (5.08 ± 1.36) months. The ratio of male to female was 9 : 10. All females were multipara and 5 of them had more than 2 cesarean deliveries. There were 12 patients with ureteral angulation and stenosis according to preoperative intravenous urography and magnetic resonance urography (MRU) and 7 patients with complete obstruction at a length of 5–7 cm, with 63.16% of angulation and stricture of the ureter and 36.84% of complete ureteral obstruction, as shown in Figure 2.  Figure 3 shows the detailed etiological distribution. 10 patients had left-sided lesions and 9 cases had right-sided lesions, as shown in Figure 4.

### 3.2. Clinical Indicators

All patients underwent psoas hitched bladder flap ureteroplasty successfully with no serious complications that occurred in the perioperative period, as given Table 1.

### 3.3. Effectiveness of the Treatment

Figure 5 shows long stenosis in the lower ureter assessed by preoperative angiography. However, the patient recovered well 2 months after surgery, as shown in Figure 6. No hydronephrosis was seen in 18 patients and only 1 patient had mild hydronephrosis (*X*^2^ = 30.421, *P* < 0.001) with no bladder ureteral stenosis, reflux, and leakage during micturition according to hilurography.

### 3.4. Safety of the Treatment

After treatment, 2 patients had low back soreness on the affected side after activities, 2 patients had hematuria which recovered without treatment, and 1 patient had a recurrent fever which recovered after antiinfection therapy (Table 2).

## 4. Discussion

Ureteral strictures pertain largely to iatrogenic injuries. The ureter is highly vulnerable to surgical apparatus damage due to its slender shape and blurred vision during surgery [13, 17–19]. Timely discovery and treatment of ureter injury facilitate the postoperative recovery and avoidance of complications. For an injured ureter part not longer than 3 cm, direct resection and reanastomosis are promising in treatment efficacy and contribute to rapid recovery. If the length of the ureteral defect is longer than half of the total length, resection of the injured site is considered unfavorable. Bladder flap ureteroplasty and pedicled omental ureteroplasty are commonly used in clinical treatments. Pedicled omental ureteroplasty is to wrap the damaged ureter by the omentum with a vascular pedicle and then transfer urine with its soft texture and ease of mobility. Because the greater omentum is highly absorbent and repairable, it can adhere to other tissues firmly. The key to the operation is to release the blood supply of the greater omentum. Since the blood supply to the greater omentum is distant from the lower end of the ureter, inadvertent manipulation may result in a cascade of adverse reactions due to insufficient blood supply to the greater omentum [20–23]. In contrast, bladder flap ureteroplasty is more effective, by directly removing a flap from the bladder wall to cover the defective ureter. Blood in this location is supplied directly by the bladder artery, with a short distance and less ischemia, and it is connected to the bladder and ureter, allowing for smoother catheterization.

With the continuous production of urine after surgery, the ureter and bladder are predisposed to various retrograde infections which are associated with persistent pain. Enrofloxacin is a third-generation quinolone antibiotic, especially for genitourinary system infections caused by sensitive bacteria, including simple and complicated urinary tract infections, bacterial prostatitis, and *Neisseria gonorrhoeae* urethritis or cervicitis (including those caused by enzyme-producing strains). It can control urinary tract infections and has a lower incidence of adverse reactions than levofloxacin. Shiduqing capsule is composed of 9 traditional Chinese medicinal herbs including Radix Scutellariae, Dictamni Cortex, *Salvia miltiorrhiza*, Cicadae Periostracum, Rehmanniae Radix, Angelicae Sinensis Radix, licorice, Poria, and Sophorae Flavescentis Radix and is mainly used for pruritus with blood deficiency and dampness in the skin. Rehmanniae Radix nourishes Yin and moistens dryness, *Salvia miltiorrhiza* activates blood circulation and eliminates blood stasis, Cicadae Periostracum evacuates wind and relieves itching, Dictamni Cortex clears heat and dampness, dispels wind, and relieves itching, and Sophorae Flavescentis Radix detoxifies. The whole formula has the efficacy of activating blood circulation, clearing heat, cooling blood, detoxifying, relieving dampness, dispelling wind, and diverting itch, which contributes to the prevention and treatment of urinary tract infection. Modern pharmacological studies have shown that Radix Scutellariae, *Salvia miltiorrhiza*, licorice, Poria, and Sophorae Flavescentis Radix have significant inhibitory effects on *Escherichia coli*, *Staphylococcus aureus*, *Staphylococcus albus*, *Pseudomonas aeruginosa*, *Streptococcus b*, *Mycobacterium avium*, *Pseudomonas aeruginosa*, *Mycobacterium typhi*, *Streptococcus avium*, and *Streptococcus b*, and Dictamni Cortex suppresses a variety of fungi. The Shiduqing capsule has anti-inflammatory, antiallergic, capillary permeability inhibition, and antihypoxia effects, and its clinical treatment efficacy for nongonococcal urethritis and cervicitis is better than that of minocycline.

In the present study, no ureteral reflux or stricture had been found assessed by intravenous pyelogram, bladder micturition, and renography two months after the surgery, demonstrating that laparoscopic bladder psoas hitch can repair lower ureteral injury up to 10 cm with less trauma and more rapid recovery compared with other ureteral reconstruction techniques. In addition, Miernik's research [23] indicated that psoas hitch might give rise to intermittent lumbago, which could be related to psoas syndrome caused by ligation of the genitofemoral nerve. Shao et al. [24] reported that 8 cases receiving psoas hitch bladder flap ureteroplasty showed no reflux or stenosis after the operation, as evidenced by the 9-year follow-up records, further supporting the feasibility and safety of this surgery.

## 5. Conclusion

To sum up, bladder flap ureteroplasty (psoas hitch) is an ideal treatment to lower ureteral injuries and strictures, which is safe and effective with less intraoperative bleeding and trauma and rapid recovery. It can reconstruct the damaged segment about 5–10 cm and ensure tension-free and continuity of the ureter.

## Figures and Tables

**Figure 1:** The pattern of bladder flap surgery with psoas hitch.

**Figure 2:** Types of ureteral diseases (%).

**Figure 3:** Causes of injury stenosis of the lower ureter (%). Note: all of the 10 patients with ureter iatrogenic injury suffered delayed diagnosis or failed open surgery.

**Figure 4:** Location of the lesion (%).

**Figure 5:** Preoperative cystography.

**Figure 6:** Cystography 2 months after operation.

**Table 1:** Statistics of clinical indicators.

Statistic index	Range	Mean value
Operative duration (min)	90.18–210.02	125.36 ± 15.38
Intraoperative blood loss (ml)	30.68–150.14	75.37 ± 11.09
Catheter extubation time (d)	5.31–11.04	7.25 ± 1.04
Hospital stay (d)	5.40–14.51	8.76 ± 1.11
Extubation time of ureteral stent (d)	28.41–90.21	46.34 ± 7.66
Follow-up time (months)	4.45–34.31	19.27 ± 1.27

**Table 2:** Statistics of postoperative adverse reactions (*n* = 19).

Postoperative adverse reactions	Cases	Incidence
Soreness of the affected side waist after activity	2	10.53
Hematuria	2	10.53
Recurrent fever	1	5.26

## Data Availability

The data generated or analyzed during this study are included within the article.
